The article "The Practices of At-Source Segregation of Household Solid Waste by the Youths in Nepal" was published in 2023. Journal: J Environ Public Health.

# The Practices of At-Source Segregation of Household Solid Waste by the Youths in Nepal

**DOI:** 10.1155/2023/5044295

**Published:** 2023-02-03

**Authors:** Ashish Khanal, Suja Giri, Prasuj Mainali

**Affiliations:** ^1^Department of Energy and Environment, Teri School of Advanced Studies, Global Research Institute and Training Center, Kathmandu, Nepal; ^2^Global Research Institute and Training Center, Kathmandu, Nepal; ^3^Jiwanta Nepal, Kathmandu, Nepal

## Abstract

Source segregation, the first important step for effective solid waste management, is practised by a handful of organizations in limited areas in Nepal. The inadequacy of source segregation and ineffective collection system in Nepal have led to maximum waste reaching the landfill site. Though several researchers have studied the role of stakeholders and the importance of youths in the waste management sector, there is a paucity of studies on the role of youths, particularly in waste segregation in Nepal. In this regard, this study was conducted to understand the at-source household waste segregation practices by youths in Nepal. The study adopted the snowball sampling technique. A structured survey questionnaire which included information on the sociodemographic status of the respondents, placement of bins, segregation practices, and satisfaction with the waste collection provider was used to elicit information from 522 youths. It was found that almost half (49.2%) of the respondents had installed two dustbins in their kitchen with 80.3% of respondents claiming to practice source segregation in their houses. The majority (75.1%) of participants were ready to pay more for improved solid waste management in their area. Also, 75.8% of respondents declared that everyone is responsible for solid waste management with fewer than 14.8% and 9.4%, stating that waste management should be the responsibility of the government and waste management service provider, respectively. The gender and source segregation was statistically significant with a *p* value of 0.007 (<0.05). However, the likelihood ratio significance showed no association between the level of education and the practice of source segregation. Hence, the source segregation practice of household solid waste was found to be satisfactory among the youths of Nepal. Thus, there should be a proper monitoring mechanism to ensure that household waste gets collected in a segregated form causing less burden on landfills.

## 1. Introduction

Global waste generation has increased from 635 million tons in 1965 to 1999 million tons in 2015 and is forecasted to reach 3539 million tons by 2050 [1]. Asia has seen a notable increase in solid waste generation due to rapid urbanization, industrialization, and economic growth since 2000 [2]. Around one-fourth of global solid waste is generated in the Asian region which is predicted to be about one-third by 2050 [3]. Unfortunately, there is no proper system of source segregation, collection, and disposal in Asian countries [4]. Apart from that, rapid population growth and urbanization have also caused an increase in the generation of household solid waste [5, 6]. Lack of skilled manpower, irregular waste collection services, inadequate equipment used for waste collection, inadequate legal provisions, and resource constraints are factors responsible for inefficient solid waste management in all developing countries [7]. Nepal, a South Asian country, is facing greater challenges with solid waste management caused due to rapid urbanization [8, 9].

The history of solid waste management in Nepal goes back to 1919 after the establishment of Safai Adda in Kathmandu [10, 11]. Though the government started waste management from their level around 100 years ago in Nepal, it is important to understand that the local authorities are not solely responsible for solid waste management [12]. Waste management is a public issue and involves the predefined role of every stakeholder. Baseline data of solid waste management in Nepal [4] show a daily waste generation of 1435 tons per day with an average per capita household waste generation rate of 170 gm/capita/day. Organic waste comprises of 66% followed by plastic (12%) and paper (9%). Another study conducted by the Central Bureau of Statistics in 2021 [13] found that the municipal waste generation in Nepal has reached 1653 tons per day with organic waste comprising of 54%. It shows that there is a high potential for recyclable extraction from the waste stream [14]. However, the waste recovery rate of Nepal is very low causing the maximum waste to reach the landfill site [15]. After the new constitution was established in 2015, Nepal has formed hundreds of new municipalities; several of which do not have formal waste management systems [16]. A huge budget is allocated every year for solid waste management in Nepal, yet the major portion of the budget is spent on street sweeping [17] giving less priority to recyclable extraction and environmentally friendly disposal of waste.

The solid waste management national policy of Nepal in 1996 had emphasized on the minimization of waste by integrating the private sector. The solid waste management act 2011 of Nepal has also focused on source segregation of waste and encouraged households to reduce, reuse, and recycle waste. It shows that the private sector is active in solid waste management in Nepal for a very long period of time. The private sector has been providing household waste collection services by charging monthly fees. Thus, it is necessary to find the experience of youth regarding the waste management service provided in their area. The willingness to pay for the solid waste management service is very much important for private sector participation in the waste management system [18]. Once the waste is segregated at the source, recyclables can be easily extracted and occupational hazards during waste separation can also be reduced [19].

Youths are important stakeholders and respond to environmental threats with better civic engagement and personal responsibility [20]. Most of the researchers agree that source segregation is very important for a better recycling system [21–24]. Waste recovery and reuse can, also, provide economic benefits to the people [25]. In this case, the role of youth is very important in creating a cultural shift towards sustainability and environmental justice [26]. Researchers from Singapore [27], Kenya [28], Egypt [29], Iran [30], Indonesia [31], India [32], and Uganda [33] have focused on the major role of youths in waste management. However, an in-depth study with a focus on source segregation has been lacking in the studies. The involvement and participation of all stakeholders are key factors for sustainable waste management [34]. Also, the role of youths (households), one of the major stakeholders of waste management, needs to be identified. Thus, this study was intended to know the source segregation practices of the youths of Nepal.

## 2. Materials and Methods

### 2.1. Population and Sample

The study was conducted on a larger youth population of Nepal where the exact current population was unknown. The last census was conducted in Nepal in 2011 [35] which categorized youths aged between 16 and 40 years old accounting for 40% of the total population (26,494,504). Based on the population projection by the Central Bureau of Statistics [36], the population of Nepal in 2021 was 30,526,143 with a youth population of 12,210,457.

Based on the population, the sample size was calculated by using the following equation [37]:

(1) $$\begin{array}{c} n=\frac{z^{2}*N*p\left(1-p\right)}{Nd^{2}+z^{2}*p\left(1-p\right)}\text{,} \end{array}$$

where *z* stands for 95% confidence level (1.96), *N* stands for total population size, *p* is the estimated population proportion, *d* stands for the margin of error, and *n* is the sample size.

As the sample size in a social survey depends on the preferred margin of error and confidence level [38], the number of respondents was 522 calculated at a 95% confidence level with a 4.3% margin of error. The sample size obtained from the mentioned equation aligns with the sample size of the table for an infinite population (>100,000) with a precision of ±5% [39]. Krejcie and Morgan [40] also confirm that the sample size of 384 is sufficient for any population of 1,000,000 or above. Hence, the sample size of 522 was enough to conduct the study among the youths of Nepal.

### 2.2. Data Collection and Analysis

The survey questionnaire was prepared on a Google form and distributed via Facebook. Facebook was purposively chosen to collect the data as it is the most popular social media in Nepal [41]. Online surveys using social media have been widely used during crises and disasters [42]. Researchers used social media to collect data for surveys and to perform analysis [43]. A snowball technique, the most commonly used technique in social science [44], was used where the respondents were asked to share it with other youths in their circle. The Google form was accessible for three weeks. The survey questionnaire included information on sociodemographic status, placement of bins, segregation practices, and satisfaction with the waste collection provider. The data collected through the online survey were automatically added to an excel sheet by the Google form. The obtained excel sheet was exported to Statistical Package for the Social Sciences (SPSS) for further analysis. The descriptive statistics including mean and frequency were calculated along with the relation and strength between the variables.

## 3. Results and Discussion

### 3.1. Demographic Details

Out of 522 respondents, 56.5% were female and 43.5% were male. Most (96.4%) of the youths were below 29 years old with only 3.6% of respondents between the age group of 30–40 years. The majority (70.3%) of respondents had passed the bachelor level of education followed by graduation (15.5%). The least (0.4%) respondents declared that they had passed the lower secondary level. Tables 1–3 show that most (66.5%) of the youth had no income.

### 3.2. Source Segregation Practice

Almost half (49.2%) of respondents had installed two dustbins in their kitchens. Also, 35.2% of respondents claimed that they had a single bin system in their kitchen with 4.8% having no bin placed inside the kitchen. 80.3% of respondents claimed that they have been practising source segregation in their houses. A study has found that the source segregation behaviour of households has drastically changed after installing the sorting equipment in the households [45]. The current study shows that the majority of Nepalese households have installed separate dustbins for separate storage of waste, and it would be comparatively easier if asked for the people to contain the source segregation of waste in their household. A question was asked whether if they would segregate the waste if asked by the waste management service provider, and the majority (94.4%) of respondents shared a positive answer. Similarly, another question was asked so as to know if the incentives would lead to better source segregation, 40.8% said that they would start segregating waste if provided with any form of incentives. Research studies conducted in Ghana [46] also found that monetary incentives act as the motivating factor for the source segregation of household solid waste. It shows that though people are concerned about the environment, they also look for financial incentives for better motivation [47]. The option could be using a lesser waste collection service fee for those households who segregate the waste and provide the waste in a segregated form to the waste management service providers. The differential user fee with leverage to the household that segregates the waste has also been shared in a study conducted in India [48]. Apart from the monetary incentives, the gender, income, attitude, type of service provider, and locality of households also affect the source segregation behaviour of the households [46].

### 3.3. Satisfaction with Waste Collection System

About 53.0% of respondents were happy with the waste management service provider in their area. The reasons for unhappiness were asked using multiple-response questions. Out of the 248 respondents, 85.5% were unhappy with the irregularities in waste collection in their area followed by the high service fees (15.7%) and bad behaviour (13.7%) from the waste collectors. Most of the waste management service providers in Nepal transfer the collected waste directly to the landfill site. There is frequent obstruction of access to the landfill which made it difficult for waste management service providers to transfer the waste to the landfill site [9]. There are several issues including financial, technical, physical, and communication obstacles which obstructs to achieve integrated SWM [49]. In such cases, the waste collection companies do not want to collect waste from the households. However, the majority (75.1%) of participants were ready to pay more for improved solid waste management in their area. It shows that when the waste management services are regular, people are, also, willing to pay more for the services rendered.

For example, in a study conducted among households in Nigeria found that people were happy to pay the waste management fee if the service was provided regularly [18]. Another study conducted among 1560 households in Ghana also found that 53.7% of the households were willing to make an additional payment for improved services [50]. A household survey conducted in Gorkha, Nepal found that the majority (67%) of people were ready to segregate the waste if the government enforces the law [51].

Female respondents (59.4%) were more active in the source segregation of household solid waste compared to males. The gender source segregation was statistically significant with a *p* value of 0.007 (<0.05). Furthermore, the phi (*φ*) value was calculated to evaluate the strength which resulted in a weak negative association (−0.12) between gender and source segregation. The finding is similar to a survey conducted on household solid waste segregation at a source in Kazakhstan which found females to be more active in waste sorting behaviour [52]. Another study conducted in Colombia also concluded that females are more active than males in terms of at-source waste segregation [53]. Women are more engaged in household chores in Nepal and more likely to deal with the daily generated household waste. Studies have found that women are likely to recycle more than men and play an important role in solid waste management at the household level [54].

When a cross tab of source segregation with education was derived, the majority (70.9%) of bachelor-level respondents were practising source segregation at their house. The expected value count for education with source segregation less than 5 was found to be 41.7% which violated our assumption (required < 20%). The likelihood ratio significance value was calculated as 0.634 which was more than 0.05 (5% confidence level). A study among the youths of Nepal found that there is no gender difference in gaining knowledge about good environmental practices [55]. Although the education of an individual helps to encourage the at-source segregation of waste [30, 56], this study did not find any association between the level of education and the practice of at-source segregation among the youths of Nepal.

## 4. Conclusion

The source segregation practice of household solid waste was found to be satisfactory among the youths of Nepal. However, the youths are not satisfied with the waste management service provided in their area. Though the majority of youths have been practising source segregation at their houses, the waste collector service provider has been collecting waste in the mixed form. The majority of youths are ready to pay more for improved waste management services. The influence of gender on source segregation was found to be statistically significant while the likelihood ratio significance showed no association between the level of education and the practice of source segregation. As there is high enthusiasm among youth regarding the source segregation of household waste, there is an urgent need for a proper monitoring mechanism from the government to ensure that the household waste gets collected in a segregated form to reduce the volume transported to the landfills.

## Figures and Tables

**Table 1:** Demographic details of the respondents.

Characteristics	*n* = 522	%
*Gender*		
Male	227	43.5
Female	295	56.5

*Education*		
Lower secondary	2	0.4
Secondary	3	0.6
Higher Secondary	56	10.7
Bachelor	367	70.3
Graduate	81	15.5
Postgraduate and above	13	2.5

*Income*		
Less than 10,000	32	6.1
10,000–30,000	75	14.4
30,000–50,000	47	9.0
50,000 and above	21	4.0
No income	347	66.5

**Table 2:** Waste segregation practices among the youths of Nepal.

Characteristics	*n*	%
*Number of bins in the kitchen*		
One	184	35.2
Two	257	49.2
More than two	56	10.7
No bins inside the kitchen	25	4.8

*Source segregation*		
Yes	419	80.3
No	103	19.7

*Segregation if asked*		
Yes	493	94.4
No	29	5.6

*Segregation if incentives*		
Yes	213	40.8
No	6	1.1
Maybe	303	58.0

*Preferred advantage for segregating waste at n* *=* *522 and 810 responses source*		
Free compost	190	36.4
Cash discount on service fee	219	42
Privilege in service provided by local government	157	30.1
Infrastructure set up in your community	244	46.7

*Waste collected separately*		
Yes	19	3.6
No	503	96.4

**Table 3:** Associations between sociodemographic characteristics and source segregation of household solid waste.

Characteristics	Source segregation (%) *n* = 522		Assumption violation (yes/no)	chi-square significance (*p* value)	Likelihood ratio	Significant (yes/no)
	Yes	No				
*Gender*						
Male	170 (40.6)	57 (55.3)	No	0.007	0.007	Yes
Female	249 (59.4)	46 (44.7)				

*Education*						
Lower secondary	1 (0.2)	1 (1.0)	Yes	0.574	0.634	No
Secondary	2 (0.5)	1 (1.0)				
Higher secondary	41 (9.8)	15 (14.7)				
Bachelor	297 (70.9)	70 (68.6)				
Graduate	67 (16.0)	14 (13.7)				
Postgraduate and above	11 (2.6)	1 (1.0)				

*Income*						
Less than 10,000	22 (5.3)	10 (9.7)	No	0.581	0.633	No
10,000–30,000	61 (14.6)	14 (13.6)				
30,000–50,000	38 (9.1)	9 (8.7)				
50,000 and above	17 (4.1)	4 (3.9)				
No income	281 (67.1)	66 (64.1)				

## Data Availability

The data used to support the findings of this study are available from the corresponding author on reasonable request.
